# Long Non-coding RNA LINC00320 Inhibits Tumorigenicity of Glioma Cells and Angiogenesis Through Downregulation of NFKB1-Mediated AQP9

**DOI:** 10.3389/fncel.2020.542552

**Published:** 2020-12-22

**Authors:** Lisha Chang, Zhe Bian, Xin Xiong, Jian Liu, Dali Wang, Fuling Zhou, Jiang Zhang, Yunhe Zhang

**Affiliations:** ^1^Department of Neurology, North China University of Science and Technology Affiliated Hospital, Tangshan, China; ^2^Department of Neurosurgery, North China University of Science and Technology Affiliated Hospital, Tangshan, China

**Keywords:** long intergenic non-coding RNA 00320, glioma, nuclear factor kappa b subunit 1, tumorigenicity, angiogenesis 3, aquaporin 9

## Abstract

The inhibitory effect of long intergenic non-coding RNA 00320 (LINC00320) in glioma cell proliferation has been proposed in a recent study. However, the mechanisms by which LINC00320 regulate aquaporin 9 (AQP9) in glioma require further exploration. Hence, this study aims to investigate effects of LINC00320 on tumorigenicity of glioma cells and angiogenesis of microvascular endothelial cells (MVECs). Expression of LINC00320 and AQP9 in glioma tissues and cells was measured by reverse transcription–quantitative polymerase chain reaction and Western blot analysis. The relationship among LINC00320, nuclear factor κB subunit 1 (NFKB1) and AQP9 was examined by RNA immunoprecipitation, dual-luciferase reporter gene, and chromatin immunoprecipitation assays. The participation of LINC00320 and AQP9 in glioma cell proliferation and MVEC angiogenesis was analyzed using gain- and loss-of-function approaches. Finally, a nude mouse orthotopic xenograft model of glioma was established to investigate the effects of LINC00320 and AQP9 on glioma growth *in vivo*. LINC00320 was under-expressed and AQP9 was over-expressed in glioma tissues. Further mechanistic investigation showed that LINC00320 downregulated AQP9 by inhibiting the recruitment of NFKB1 to the promoter region of AQP9. LINC00320 overexpression or AQP9 silencing inhibited the proliferation of glioma cells and angiogenesis of MVECs. Also, upregulation of LINC00320 restrained tumor growth and angiogenesis in xenograft mice by downregulating AQP9. Taken together, LINC00320 acts as a tumor suppressor in glioma, thus presenting a novel therapeutic target.

## Introduction

In 2018, there were 296,851 newly diagnosed cases of malignancies of the brain and nervous system reported worldwide, which brought very high mortality (Bray et al., 2018). Gliomas are primary brain malignancies, which are derived from neuroglial stem or progenitor cells (Weller et al., 2015). Ionizing radiation, inherited genotype, and smoking are among the known risk factors for brain cancers including glioma (Savage, 2018). Although several therapeutic approaches including surgery, irradiation, and temozolomide therapy bring some remission in glioma treatment, tumor relapse is still inevitable and unrelenting, eventually causing patient death (Sanai and Berger, 2018). Advancement in molecular profiling contributes to obtaining a comprehensive characterization of the genetic and epigenetic alterations in gliomas by revealing new biomarkers that can guide individualized treatments (Reifenberger et al., 2017).

At present, an abundance of identified long non-coding RNAs (lncRNAs) are known to play indispensable roles in the pathogenesis and biological processes of glioma, such as stemness, angiogenesis, and drug resistance (Peng et al., 2018). Long intergenic non–protein-coding RNAs, a class of ncRNA species exceeding 200 nucleotides in length, cover more than half of lncRNA transcripts and share characteristics with other lncRNA transcripts in humans (Ransohoff et al., 2018). Of note, Tian et al. (2019) have provided detailed data confirming the function and presenting a mode of action for LINC00320 in glioma progression whereby LINC00320 exerts inhibitory effects on glioma cell proliferation by restraining the Wnt/β-catenin signaling through segregating β-catenin and transcription factor 4 (TCF4). Additionally, it has recently been acknowledged that lncRNAs are critical regulators of the transcriptional process, which can bind to DNA binding proteins that are transcription factors (TFs; Long et al., 2017). In general, TFs control the transcription of genes and also underlie different aspects of human physiology and diseases (Lambert et al., 2018). One notable TF, nuclear factor κB (NF-κB) subunit 1 (NFKB1), has been suggested to crucially function in the progression of human cancers (Concetti and Wilson, 2018). Through the computational lncRNA–TF gene prediction based on the LncMap database, we proposed in this study a possible interaction among LINC00320, NFKB1, and aquaporin 9 (AQP9). The AQP water channels have been highlighted as important regulators in nervous system and hold great potential as promising therapeutic targets for brain disorders (Xu et al., 2017). AQP9 is a water channel protein with limited expression in normal brain, but an increased level of AQP9 is seen in glioma tissues and cells (Fossdal et al., 2012; Jelen et al., 2013). Hence, we speculated that LINC00320 might bind to NFKB1 to regulate the transcription of AQP9, which might possibly be involved in the progression of glioma.

In the present study, we aim to validate the proposed interaction whereby LINC00320 regulates the expression of AQP9 by binding to NFKB1 and altering transcription. In addition, we investigated the effects of LINC00320 on glioma development and tumor angiogenesis and provided evidence that LINC00320 may be a potential therapeutic target for glioma treatment.

## Materials and Methods

### Ethics Statement

The current study was performed with the approval of the Clinical Trial Ethics Committee of North China University of Science and Technology Affiliated Hospital (reference number of the approval: 201402006). All patients and their families in the experiment gave informed consent to the experiment and signed informed consent. The animal experiments were approved by the Experimental Animal Ethics Committee (reference number of the approval: 201501003) and strictly adhered to the principle to minimize the pain and discomfort to experimental animals.

### Microarray-Based LncRNA Expression Profiling

The microarray data GSE104291 related to glioma was downloaded from the Gene Expression Omnibus database^1^, which consists of 24 cancer tissue samples and 2 normal tissue samples. With the use of the Limma package and |log2FoldChange| >4 and *p* < 0.05 set as the threshold, we obtained the differentially expressed lncRNAs related to glioma and the expression of LINC00320 in glioma cells. Next, LINC00320 was predicted using the LncMap^2^ database, and the possible relationship between lncRNA, TFs, and genes was identified.

### Study Subjects

Eighty-three patients who were diagnosed with glioma by pathological examination and underwent surgery at North China University of Science and Technology Affiliated Hospital from June 1, 2015, to May 31, 2016, were enrolled in the study. Among them, there were 44 males and 39 females of mean age 39.5 ± 18.0 years (range, 12–78 years). Those patients were divided into four subgroups based on the World Health Organization classification, including 25 cases of grade I, 21 cases of grade II, 24 cases of grade III, and 13 cases of grade IV. No patient had received radiotherapy and/or chemotherapy before surgery. 10 normal brain tissues obtained during intracranial decompression surgery from patients with traumatic brain injury (Fei et al., 2018) were used as the control group, consisting of seven males and three females, of mean age 36.2 ± 19.0 years (range, 14–68 years). The 3-year overall survival was calculated using the Kaplan–Meier method.

### Reverse Transcription–Quantitative Polymerase Chain Reaction

Total RNA was extracted using TRIzol kit (15596026; Invitrogen, Carlsbad, CA, United States), and cDNA was generated from the extracted RNA using reverse transcription (RT) kit (RR047A, Takara, Tokyo, Japan). An SYBR Premix EX Taq kit (RR240A, Takara) was adopted for real-time quantitative polymerase chain reaction (qPCR) in a real-time PCR instrument (ABI7500; Applied Biosystems, Foster City, CA, United States). Each experiment was conducted in triplicate. The primers generated by Sangon (Shanghai, China) are depicted in Table 1. After recording of Ct values, the expression of target genes was calculated by the 2^–ΔΔCt^ method standardized by β-actin.

**TABLE 1:** Primer sequences for reverse transcription quantitative polymerase chain reaction.

**Gene**	**Sequence**
AQP9	F: 5′-CGGCATTTGTACAGTCAGAGACTC-3′
	R: 5′-AATGCGTTCGCCAGAGATAGATAC-3′
NFKB1	F: 5′-GGCAGCACTACTTCTTGACC-3′
	R: 5′-CAGCAAACATGGCAGGCTAT-3′
LINC00320	F: 5′-GACTCCTTTGGGAGACCAGTG-3′
	R: 5′-AGGTCACAGGGGATTTGATGG-3′
β-Actin	F: 5′-CGCACCACTGGCATTGTCAT-3′
	R: 5′-TTCTCCTTGATGTCACGCAC-3′

*AQP9, aquaporin 9; NFKB1, nuclear factor κB subunit 1; LINC00320, long intergenic non-coding RNA 320; F, forward; and R, reverse.*

### Western Blot Analysis

The sample stored in the −80°C freezer was thawed and then added with tissue lysis buffer to prepare a homogenate using a Teflon-glass piston. After high-speed centrifugation, the supernatant was collected and then mixed well with the loading buffer, heated, and stored in a freezer at −20°C. The protein was subsequently separated using separation and spacer gels and transferred onto a nitrocellulose membrane. After skimmed milk blocking, the membrane was probed with rabbit polyclonal antibodies (Abcam Inc., Cambridge, United Kingdom) to AQP9 (1:5,000, ab15127) and vascular endothelial growth factor (VEGF; 1:1,000, ab53465, Abcam), rabbit antibody to NFKB1 (1:500, ab32360), and rabbit antibodies (Abcam) to phosphorylated NFKB1 (1:500, ab28849), CD31 (1:500, ab28364), matrix metalloproteinase-2 (MMP-2; 1:1,000, ab92536), and MMP-9 (1:5,000, ab76003) overnight at 4°C. Next, the membrane was reprobed with horseradish peroxidase–labeled goat polyclonal antibody to immunoglobulin G (IgG; HA1003, Shanghai Research Biotechnology Co., Ltd., Shanghai, China) and rabbit antibody to IgG (1:2000, ab6721, Abcam). After washing, the membrane was developed with enhanced chemiluminescence reagent (ECL808-25; Biomiga, San Diego, CA, United States), washed, air-dried, and scanned with a gel image analyzer. The ratio of the gray value of the target band to glyceraldehyde-3-phosphate dehydrogenase (GAPDH) was calculated by a four-star image processing system. The experiment was repeated three times independently.

### Cell Culture and Transfection

Glioma cell lines including LN229 (CRL-2611), U87 (HTB-14), U251, and T98G (CRL-1690; all from American Type Culture Collection, Manassas, VA, United States) and human normal brain glial cell line HEB were used in this study. Then, the expression of LINC00320 in these cells was determined by RT-qPCR, and the cell line presenting the lowest LINC00320 expression was selected for subsequent experiments. Cells were cultured in Dulbecco modified eagle medium (DMEM) from Gibco Company (Grand Island, NY, United States) containing 10% fetal bovine serum, 100 U/mL penicillin (Sigma, St. Louis, MO, United States), 100 U/mL streptomycin (Sigma), and 2 mM of L-glutamic acid (Sigma). The medium was renewed every 2 to 3 days. When the cells reached 80% to 90% confluence, cells were passaged. The cells in the logarithmic growth phase were transfected with plasmids of overexpressing LINC00320 (oe-LINC00320), oe-negative control (NC), oe-LINC00320 + oe-NC, oe-LINC00320 + oe-NFKB1, or oe-LINC00320 + oe-AQP9.

The aforementioned plasmids were all purchased from Dharmacon (Lafayette, CO, United States). The glioma cells were seeded in a six-well plate at a density of 3 × 10^5^ cells/well. When the cells reached 80% confluence, the cells were cultured with 500 μL of DMEM. Next, 10 μL of Lipofectamine^TM^ 2000 (Takara) was diluted with 250 μL of serum-free MEM (Invitrogen) and incubated at room temperature for 5 min. After that, 4.0 μg of recombinant plasmid was added to the aforementioned 250 μL of serum-free MEM containing 10 μL Lipofectamine^TM^ 2000, followed by 20-min incubation at room temperature. Then, 50 μL of recombinant plasmid-Lipofectamine complex was added to each cell culture well. The plate was gently shaken and mixed, and the cells were cultured in a 37°C incubator with 5% CO_2_. The cells were cultured with renewed medium 6 h after incubation and harvested 36 to 48 h after transfection. Oligonucleotides for cell transfection are listed in Table 2.

**TABLE 2:** Oligonucleotides for cell transfection.

**Gene**	**Oligonucleotides**
AQP9	F: 5′-ccgaattcATGCAGCCTGAGGGAGCA-3′
	R: 5′-cgggtaccCTACATGATGACACTGAGTTCATATTTC-3′
NFKB1	F: 5′-ccgaattcATGGCAGAAGATGATCCATATTT-3′
	R: 5′-cgggtaccCTAAATTTTGCCTTCTAGAGGTCC-3′
LINC00320	F: 5′-ccgaattcACTGTGTGATTTTTGTTCTTTAGTAGA-3′
	R: 5′-cgggtaccAATAATACAGTCATCCACAGATTTTAT-3′

*AQP9, aquaporin 9; NFKB1, nuclear factor κB subunit 1; LINC00320, long intergenic non-coding RNA 320; F, forward; and R, reverse.*

### Cell Counting Kit 8

The glioma cells were incubated in a 96-well plate and arranged into four groups. Each well was added with 10 μL cell counting kit 8 (CCK-8) reagent (Dojindo Laboratories, Kumamoto, Japan) before 6, 12, 24, and 48 h of cells being incubated at 37°C. The absorbance (A450) value of each well was measured by a Multiskan GO microplate reader (Thermo Fisher Scientific Inc., Waltham, MA, United States). Cell viability was subsequently calculated with the formula: cell viability (%) = absorbance value in the experimental group/absorbance value in the blank group × 100%.

### Trypan Blue Staining

When at the logarithmic growth phase, cells were trypsinized. With the concentration adjusted to 3 × 10^7^ cells/L, cells were incubated in a 96-well plate at 37°C with 5% CO_2_ overnight. The plate was placed in an incubator at 37°C with 5% CO_2_ after 4-h adherent cell transfection with corresponding plasmids or inhibitor. Cells were trypsinized after transfection for 72 h and stained with trypan blue to count the number of dead cells.

### RNA-Binding Protein Immunoprecipitation Experiment

RNA-binding protein immunoprecipitation (RIP) was operated using Magna RIP^TM^ RNA Binding Protein Immunoprecipitation Kit (MiLople, Billerica, MA, United States) and 2 μg NFKB1 antibody (sc-166588; Santa Cruz Biotechnology, Dallas, Texas, United States) in strict accordance with the instructions. In brief, after lysing in RIP lysis buffer, cell lysate was incubated with A + G magnetic beads coated with antibody to NFKB1. The normal antibody to IgG (microwell) was regarded as negative control (NC), and antibody to snRNP70 was used as a positive control (MiL microwell). The immunoprecipitated RNA was obtained by culturing the samples with proteinase K. The immunoprecipitated RNA was detected by RT-qPCR. The primer sequences of LINC00320 for RT-qPCR were as follows: forward primer 5′-ATGACAGTTGGCAATGCAGC-3′ and reverse primer 5′-ATGACAGTTGGCAATGCAGC-3′.

### Dual-Luciferase Reporter Gene Assay

Target genes of TF NFKB1 were predicted by bioinformatics website. Primers containing restriction endonuclease sites *Mlu*I and *Xho*I were designed on polyclonal sites of pGL3-basic vector. Double-enzyme digestion was conducted on AQP9 promoter fragment containing restriction sites and pGL3-basic vector using *Mlu*I and *Xho*I. The products were treated with T4 ligase and transformed into DH5α competent cells. The positive cloning was screened out, followed by identification through sequencing and double-enzyme digestion. A recombinant vector of AQP9 wild type (WT) was obtained. The correctly sequenced luciferase reporter plasmid was co-transfected into HEK293T cells with oe-NFKB1 and oe-NC, respectively. After 48-h transfection, the cells were lysed. With Renilla luciferase as internal reference, luciferase activity was measured using a luciferase reporter assay kit (K801-200; Biovision, Milpitas, CA, United States) and a dual-luciferase reporter gene assay system (Promega, Madison, WI, United States). The ratio of relative light unit of firefly luciferase to that of Renilla luciferase was used to compare the luciferase activity of target reporter genes.

### Chromatin Immunoprecipitation

Glioma cells were incubated into 10-cm culture dishes at 10^6^ cells per well. The cells were fixed with approximately 1% formaldehyde solution before 5-min incubation at room temperature. The cells were subsequently ultrasonicated, and the DNA was sheared. Next, the DNA was precipitated by adding NFKB P65 antibody (2 μg, sc-166588; Santa Cruz). Next, DNA protein was precipitated by supplementing protein agarose/sepharose. After proteinase K treatment and de–cross-linking, the DNA was purified. Subsequently, RT-qPCR was conducted to detect the immunoprecipitated DNA. The primer sequence of the AQP9 promoter I region was forward: 5′-CTCAGTGTCATCATGTAGTG-3′ and reverse: 5′-GACTATCGTCAAGATGCCG-3′. The chromatin immunoprecipitation (ChIP) efficiency was detected following ultrasonical cleavage and purification of chromatin fragments (input DNA). The PCR system comprised 12.5 μL rTaq or SYBR Premix Ex Taq^TM^II; 1 μL forward primer and 1 μL reverse primer (10 μmol/L); and 3 μL DNA template, with the addition of sterilized distilled water to reach a total volume of 25 μL. The amplification conditions were as follows: predenaturation at 95°C for 10 min, denaturation at 95°C for 60 s, and extension 72°C for 30 s, 40 cycles in total. The results were expressed as% input = 2 (Ct_Input_-Ct_ChIP_) × input dilution factor × 100.

### Immunofluorescence for Detection of NFKB1

After administration and medium renewal, cells were fixed with 20 g/L paraformaldehyde for 10 min before 20-min culture with 0.5% Triton X-100 and 30-min sealing with 5% bovine serum albumin (BSA). Then, rabbit anti–human monoclonal antibody to NFKB1 (1:100, ab32360; Abcam) was added before overnight cell culture at 4°C. Then, 1-h cell reprobing was conducted with secondary antibody (1:200) at room temperature, followed by 5-min nucleus staining with 4′,6-diamidino-2-phenylindole under condition void of light. After sealing in anti-fluorescence quenching agent, the sample was observed under a fluorescent inverted microscope.

### Tube Formation Assay *in vitro*

The glioma cells were co-cultured with human microvascular endothelial cells (MVECs), HMEC-1, to detect the tube formation ability of the microvascular endothelium. The Matrigel was frozen and thawed overnight at 4°C. Then, 75 μL of Matrigel was added to each well in a precooled 96-well plate before 60-min culture at 37°C. The suspension of HMEC-1 (HCCL-013; Shanghai Yanjin Technology Co., Ltd., Shanghai, China) was plated to the 96-well plate at 2.5 × 10^4^ cells/well. After the cells were adhered to the walls, the culture solution was renewed with the supernatant of the glioma cell line after transfection, followed by further incubation. After 4–6 h, images of five randomly selected fields were captured using a microscope (Olympus, Tokyo, Japan) with 100 × magnification and analyzed using ImageJ software.

### Nude Mouse Orthotopic Xenograft Model of Glioma

Thirty BALA/C nude mice aged 6 weeks and weighing 18–22 *g* (gender unlimited), purchased from Hunan SLAC Laboratory Animal Co., Ltd. (Hunan, China), were acclimated in specific pathogen free environment. The U87 cells stably transfected with oe-NC, oe-LINC00320 + oe-NC, or oe-LINC00320 + oe-AQP9 were dispersed into cell suspension. The nude mice were subcutaneously injected with U87 cell suspension (*n* = 10 mice/treatment). The tumor growth was observed every 2 to 3 days, and the tumor size was measured using Vernier calipers. After the experiment, the mice were euthanized via anesthesia overdose. The tumors were collected, followed by photographing and weighing. The volume of the transplanted tumors was calculated as follows: *V* (mm^3^) = (*A* × *B*^2^)/2 (*A* representing the long diameter, and *B* the short diameter).

### Immunohistochemistry for Detection of CD31 Protein

The specimen was fixed with 10% formaldehyde before preparation of 4-μm paraffin-embedded sections. The sections were then positioned in a 60°C thermostatically controlled bath for 1 h, followed by conventional xylene dewaxing and gradient alcohol rehydration. Following retrieval with 0.1 M sodium citrate, the sections were boiled for 20 min and allowed to cool down. After that, the sections were treated with 3% catalase for 15 min. After three washes with phosphate-buffered saline (PBS; 0.2 M; pH 7.4; 5 min each), 30-min section culture was performed with 5% BSA at 37°C. Thereafter, the sections underwent overnight incubation with rabbit antibody to CD31 (1:500, ab28364, Abcam) at 4°C. Following 30-min reprobing with biotinylated goat anti–rabbit IgG (1:2000, ab205718, Abcam) at 37°C, the sections were developed by diaminobenzidine (DA1010, Beijing Solarbio Science & Technology Co., Ltd., Beijing, China) in a darkened room for 8 min. The sections were counterstained with hematoxylin, dehydrated, cleared, sealed, and observed under a biological microscope (XSP-36; Boshida Optical Instrument Co., Ltd., Shenzhen, China). Positive expression appeared as yellow/brown–yellow particles in cell membrane or cytoplasm. We then counted 100 cells in each of five randomly selected fields. Negative was defined as the number of positive cells < 5%, and positive was defined as the number of positive cells ≥ 5%.

### Terminal Dexynucleotidyl Transferase-Mediated 2′-Deoxyuridine 5′-Triphosphate Nick End Labeling (TUNEL) Assay

The 4-μm sections were subjected to TUNEL assay for cell apoptosis detection in the light of the manual of a commercially provided kit (Roche Life Science, Basel, Switzerland). Sections were conventionally dewaxed and hydrated, and endogenous peroxidase was removed. The tissue proteins were discarded through detachment using proteinase K at 37°C for 20 min. Following treatment using 0.1% Triton, TUNEL reaction solution was added for 1-h incubation in a wet box at 37°C, with 10 mM PBS (pH 7.4) used for rinsing in the above steps. We set PBS as NC, and positive control groups were set. The sections were sealed by neutral resin and glycerol before observation and photographing under an inverted fluorescence microscope. The presence of brown-stained grains was indicative of apoptotic cells.

### Statistical Analysis

Statistical analysis was processed using SPSS 21.0 software (IBM, Armonk, NY, United States), with *p* < 0.05 as statistically significant. All experimental results were scored by two observers with the double-blinded method. Image quantification analysis was conducted by ImageJ software. The measurement data were summarized as mean ± standard deviation. Comparison between two groups was analyzed by independent-sample *t* test, and data among multiple groups were analyzed by one-way analysis of variance (ANOVA), followed by Tukey multiple-comparisons posttest. Statistical analysis at different time points between two groups was achieved with independent-sample ANOVA. The relationship between high and low expression of LINC00320 and overall survival in glioma tissues (log-rank test) was analyzed by Kaplan–Meier.

## Results

### LINC00320 Is Poorly Expressed While AQP9 Is Highly Expressed in Glioma Tissues

Analysis of the gene expression dataset GSE104291 revealed 359 differentially expressed genes in glioma, of which 91 genes were highly expressed and 268 were poorly expressed (Figure 1A). Previous work has indicated that LINC00320 that is localized in the nucleus inhibits the proliferation of glioma cells *in vivo* and *in vitro* (Tian et al., 2019). Our differential analysis results indicated that LINC00320 was downregulated in gliomas (Figure 1B). To further investigate the regulatory mechanism of LINC00320 in glioma, we employed the LncMap database to predict the target gene of LINC00320. Existing literature has shown that AQP9 was downregulated in normal brain, while being highly expressed in human gliomas (Jelen et al., 2013). Therefore, we selected AQP9 as an entry point to investigate the possible TFs involved in the process whereby LINC00320 regulated AQP9. Through the prediction results from the LncMAP database, we found that the TF NFKB1 was involved in the regulation of LINC00320 (Table 3). Therefore, we hypothesized that LINC00320 may inhibit the proliferation of glioma cells by regulating AQP9 expression via NFKB1.

**FIGURE 1:** LINC00320 was expressed at a low level, and AQP9 was expressed at a high level in glioma tissues. **(A)** Volcano map representing differentially expressed lncRNAs related to glioma. The abscissa indicates log fold change, and the ordinate indicates log10 *p* value. Each point in the figure represents a gene, the red dots indicate upregulated genes, and the green dots indicate downregulated genes. **(B)** The expression of LINC00320 in gliomas and normal samples evaluated by differential analysis. **(C)** The expression of LINC00320 in glioma (*n* = 83) and normal brain tissues (*n* = 10) determined using RT-qPCR normalized to β-actin. **(D)** Overall survival curve of patients with glioma regarding the expression pattern of LINC00320 plotted using Kaplan–Meier method. **(E)** The mRNA expression of AQP9 in glioma (*n* = 83) and normal brain tissues (*n* = 10) detected using RT-qPCR normalized to β-actin. **(F)** AQP9 protein expression normalized to GAPDH in glioma (*n* = 83) and normal brain tissues (*n* = 10) measured by Western blot analysis. *p < 0.05 vs. normal brain tissues. Data were expressed as mean ± standard deviation, and independent-sample *t* test was used for data analysis. Kaplan–Meier was used to analyze the relationship between expression of LINC00320 in glioma tissues and overall survival of patients (log-rank test).

**TABLE 3:** Possible participation of LINC00320, NFKB1, and AQP9 in glioma predicted by LncMap database.

**Cancer type**	**LncRNA symbol**	**TF symbol**	**Gene symbol**	**Mediated pattern**
GBM	LINC00320	NFKB1	AQP9	+++

*LncRNA, long non-coding RNA; TF, transcription factors; GBM, glioblastoma multiforme; LINC00320, long intergenic non–protein-coding RNA 320; NFKB1, nuclear factor κB subunit 1; and AQP9, aquaporin 9.*

To detect LINC00320 expression in glioma, LINC00320 expression in 83 glioma tissues and 10 normal brain tissues was measured by RT-qPCR. As depicted in Figure 1C, LINC00320 was downregulated in glioma tissues vs normal brain tissues (*p* < 0.05). Subsequent results showed that LINC00320 expression was correlated with pathological grade and metastasis of glioma (Table 4). The median value of LINC00320 expression (0.230) was taken as the cutoff point for classifying the patients into high and low expression groups, and the survival rate was analyzed using Kaplan–Meier method. The results shown in Figure 1D revealed that patients with glioma in the low expression group exhibited poor overall survival. RT-qPCR and Western blot analysis showed that, compared with normal brain tissues, mRNA and protein expression of AQP9 in glioma tissues were much higher (*p* < 0.05; Figures 1E,F). Taken together, LINC00320 was downregulated, but AQP9 was upregulated in glioma tissues.

**TABLE 4:** Relationship between the expression of LINC00320 and clinical characteristics of patients with glioma.

**Clinical characteristics**	**LINC00320**		***p***
	**High expression**	**Low expression**	
Gender			0.511
Male	21	23	
Female	22	17	
Age (years)			0.123
<45	29	20	
≥45	14	20	
WHOstage			0.008
I, II	30	16	
III, IV	13	24	
Tumor size			0.028
≤3 cm	26	14	
>3 cm	17	26	
Metastasis			0.023
No	22	10	
Yes	21	30	

*The table indicates statistical results from χ^2^ analysis. LINC00320, long intergenic non–protein-coding RNA 320; and WHO, World Health Organization.*

### LINC00320 Is Expressed at a Low Level in Glioma Cells

Long intergenic non-coding RNA 00320 expression in normal human glial cell line HEB and four glioma cell lines LN229, U87, U251, and T98G was determined by performing RT-qPCR. The results revealed that LINC00320 was downregulated in glioma cells compared with that in HEB cells, and it presented the lowest expression in U87 cells, which were chosen for the following experiments (*p* < 0.05; Figure 2).

**FIGURE 2:** LINC00320 was expressed poorly in glioma cells. LINC00320 expression in HEB, LN229, U87, U251, and T98G cell lines detected using RT-qPCR normalized to β-actin. *p < 0.05 vs. HEB cell line. Data were expressed as mean ± standard deviation, and comparisons among multiple groups were conducted by one-way ANOVA, followed by a Tukey multiple-comparisons posttest. The experiment was repeated three times independently.

### Upregulation of LINC00320 Inhibits Glioma Cell Proliferation and MVEC Angiogenesis

To test the transfection efficiency of LINC00320, NFKB1, and AQP9 in glioma cells, RT-qPCR was conducted in U87 cells. LINC003200 expression was increased in oe-LINC00320–transfected U87 cells, NFKB1 expression was elevated in oe-NFKB1–transfected U87 cells, and AQP9 expression was upregulated in oe-AQP9–transfected U87 cells (*p* < 0.05; Figure 3A). To avoid the effect of transfection on U87 cell death, trypan blue staining was performed to identify cell death in each group. Results showed that U87 cell death rate did not differ significantly in cells treated with oe-NC when compared with cells without any treatment (Supplementary Figure 1), suggesting that transfection of blank plasmids did not influence cell death. To examine the growth of cells, we measured the viability of U87 cells by CCK-8 assay, finding that delivery of oe-NC had no significant effect on U87 cell viability compared with U87 cells without any treatment, indicating that U87 cell survival is unaffected by transfection of control plasmids. Moreover, the viability of U87 cells transfected with oe-LINC00320 was reduced, whereas those transfected with oe-NFKB1 or oe-AQP9 exhibited higher cell viability compared to oe-NC–transfected cells (*p* < 0.05; Figure 3B). Furthermore, the number of tube branches in oe-LINC00320–transfected cells was reduced (*p* < 0.05; Figure 3C). Additionally, Western blot analysis manifested that VEGF, CD31, MMP-2, and MMP-9 expression was decreased in the cells after transfection with oe-LINC00320 (*p* < 0.05; Figures 3D–G). These results indicated that upregulation of LINC00320 could inhibit the proliferation of glioma cells and angiogenesis of MVECs.

**FIGURE 3:** Overexpressed LINC00320 impeded glioma cell proliferation and MVEC angiogenesis. **(A)** The expression of LINC00320, NFKB1, or AQP9 in glioma cells transfected with oe-LINC00320, oe-NFKB1, or oe-AQP9 detected using RT-qPCR normalized to β-actin. **(B)** The growth of cells transfected with oe-LINC00320 measured using CCK-8 assay. **(C)** The cellular tube formation in MVECs upon co-culture with glioma cells transfected with oe-LINC00320 (100×; scale bar = 10 μm). **(D)** Expression of angiogenesis-related VEGF protein in MVECs upon co-culture with glioma cells transfected with oe-LINC00320 normalized to GAPDH measured by Western blot analysis. **(E)** Expression of angiogenesis-related CD31 protein in MVECs upon co-culture with glioma cells transfected with oe-LINC00320 normalized to GAPDH measured by Western blot analysis. **(F)** Expression of angiogenesis-related MMP-2 protein in MVECs upon co-culture with glioma cells transfected with oe-LINC00320 normalized to GAPDH measured by Western blot analysis. **(G)** Expression of angiogenesis-related MMP-9 protein in MVECs upon co-culture with glioma cells transfected with oe-LINC00320 normalized to GAPDH measured by Western blot analysis. *p < 0.05 vs. cells transfected with oe-NC. Data were expressed as mean ± standard deviation and data between two groups were analyzed by independent-sample *t* test. Data between two groups at different time points were compared by repeated-measures ANOVA. The experiment was repeated three times independently.

### LINC00320 Downregulates the Expression of AQP9 via Recruiting NFKB1 to the Promoter Region of AQP9

To verify the functional regulatory mechanism of LINC00320, the binding of LINC00320 to NFKB1 protein was tested by performing a RIP assay. The results showed that LINC00320 enrichment was increased in the NFKB1 group as compared with the IgG group (*p* < 0.05; Figure 4A). RT-qPCR showed that overexpression of LINC00320 significantly decreased NFKB1 expression (Figure 4B, *p* < 0.05). Western blot analysis and immunofluorescence revealed diminished NFKB1 phosphorylation in response to overexpressed LINC00320, suggesting that NFKB1 phosphorylation was suppressed and that NFKB1 was mainly localized in the nucleus (Figures 4C,D; *p* < 0.05). In addition, Western blot analysis depicted that AQP9 expression and extent of NFKB1 phosphorylation were much higher in U87 cells than in HEB cells (*p* < 0.05; Figure 4E). Next, the binding of NFKB1 to the promoter region of AQP9 gene was predicted by the JAPAR database^3^ (Supplementary Table 1) and further determined by dual-luciferase reporter gene assay. The results showed that overexpression of NFKB1 significantly increased the luciferase activity of AQP9-WT (*p* < 0.05; Figure 4F), while AQP9-mutant expression remained unaffected after oe-NFKB1 transfection (*p* > 0.05). ChIP reported that the level of AQP9 promoter pulled down by NFKB1 antibody was higher than that pulled down by IgG (*p* < 0.05; Figure 4G), suggesting that NFKB1 could bind to the promoter region of the AQP9 gene. However, the level of AQP9 promoter pulled down by NFKB1 antibody was reduced after LINC00320 overexpression (Figure 4H). Finally, after transfection with oe-LINC00320 + oe-NC, oe-LINC00320 + oe-NFKB1, or their corresponding controls in U87 cells, RT-qPCR documented that overexpression of LINC00320 resulted in reduced expression of AQP9 (*p* < 0.05), while the inhibited AQP9 expression was rescued upon co-transfection with oe-LINC00320 and oe-NFKB1 (*p* > 0.05; Figure 4I). The aforementioned results indicate that LINC00320 decreased the expression of AQP9 by inhibiting the recruitment of NFKB1 to the promoter region of AQP9.

**FIGURE 4:** LINC00320 reduced the expression of AQP9 via inhibiting NFKB1. **(A)** The binding of LINC00320 to NFKB1 protein confirmed by RIP assay. **(B)** Expression of NFKB1 mRNA in response to overexpressed LINC00320 determined by RT-qPCR normalized to β-actin. **(C)** Expression of NFKB1 protein in response to overexpressed LINC00320 normalized to GAPDH determined by Western blot analysis. **(D)** Expression of NFKB1 protein in response to overexpressed LINC00320 detected by immunofluorescence. **(E)** The expression of AQP9 protein and extent of NFKB1 phosphorylation in HEB cells and glioma cells U87 normalized to GAPDH measured by Western blot assay. **(F)** The binding of NFKB1 to the promoter region of gene AQP9 confirmed by dual-luciferase reporter gene assay. **(G)** The binding of NFKB1 to the promoter region of gene AQP9 confirmed by ChIP assay. **(H)** The binding of NFKB1 to the promoter region of gene AQP9 in response to overexpressed LINC00320 confirmed by ChIP assay. **(I)** The expression of AQP9 in transfected cells determined by RT-qPCR normalized to β-actin. *p < 0.05 vs. IgG, HEB cells, or oe-NC group. Data were expressed as mean ± standard deviation, and data between two groups were analyzed by independent-sample *t* test. Data among multiple groups were analyzed by one-way ANOVA, followed by a Tukey multiple-comparisons posttest. The experiment was repeated three times independently.

### Upregulation of LINC00320 Hinders Glioma Cell Proliferation and MVEC Angiogenesis via Downregulation of AQP9

Aquaporin 9 expression in glioma cells was determined by RT-qPCR after transfection with oe-LINC00320 + oe-NC or oe-LINC00320 + oe-AQP9. Results showed that AQP9 expression was significantly reduced, and LINC00320 expression was elevated in glioma cells transfected with oe-LINC00320 + oe-NC in contrast to those transfected with oe-NC. On the other hand, LINC00320 expression was unaffected, whereas AQP9 expression was increased in U87 cells upon transfection with oe-LINC00320 + oe-AQP9 as compared to the effects of transfection with oe-LINC00320 + oe-NC (both *p* < 0.05; Figure 5A). The results obtained from CCK-8 and tube formation assays displayed that U87 cell viability was lowered (Figure 5B), and the number of tube branches in MVECs was reduced (Figure 5C) upon co-transfection with oe-LINC00320 and oe-NC compared with oe-NC transfection (*p* < 0.05). Moreover, those reductions induced by LINC00320 overexpression were neutralized by restoration of AQP9 expression. Next, Western blot analysis clarified that VEGF and CD31 protein expression was decreased by LINC00320 overexpression, which was rescued by restoration of AQP9 expression (all *p* < 0.05; Figures 5D,E). The above results demonstrated that LINC00320 inhibited the expression of AQP9, thereby inhibiting the growth of glioma cells and angiogenesis of MVECs.

**FIGURE 5:** LINC00320 overexpression disrupted glioma cell viability and MVEC angiogenesis by inhibiting the expression of AQP9. **(A)** The expression of LINC00320 and AQP9 in glioma cells determined by RT-qPCR normalized to β-actin. **(B)** The growth of glioma cells assessed using CCK-8 assay. **(C)** The tube formation in MVECs upon co-culture with transfected glioma cells (100×, scale bar = 10 μm). **(D)** Expression of angiogenesis-related VEGF protein normalized to GAPDH in MVECs upon co-culture with transfected glioma cells measured by Western blot analysis. **(E)** Expression of angiogenesis-related CD31 protein normalized to GAPDH in MVECs upon co-culture with transfected glioma cells measured by Western blot analysis. *p < 0.05 vs. cells transfected with oe-NC, ^#^*p* < 0.05 vs. cells co-transfected with oe-LINC00320 and oe-NC. Data were expressed as mean ± standard deviation, and comparisons among multiple groups were conducted by one-way ANOVA, followed by a Tukey multiple-comparisons posttest. The experiment was repeated three times independently.

### Upregulation of LINC00320 Inhibits Tumor Growth and Angiogenesis by Downregulating AQP9 Expression

To determine the roles of LINC00320 and AQP9 in tumorigenicity of glioma cells, the growth of the tumors in nude mice was assessed by injection with the stably transfected cells. The volume and weight of tumors of mice injected with LINC00320-overexpressed cells were reduced, which was neutralized by further overexpression of AQP9 (*p* < 0.05; Figures 6A–C). To elucidate that LINC00320 regulated angiogenesis *in vivo* by regulating the expression of AQP9, we measured VEGF expression by Western blot analysis and CD31 expression by immunohistochemistry (IHC). VEGF expression in mice was potently decreased by overexpression of LINC00320 (*p* < 0.05), whereas this decrease was normalized by restoration of AQP9 (Figures 6D,E). The number of microvessels was reduced by overexpression of LINC00320 (*p* < 0.05), but this reduction was counteracted by restoration of AQP9 (Figures 6F,G). According to TUNEL assay results, cell apoptosis rate was elevated in the presence of oe-LINC00320, yet further addition of oe-AQP9 decreased the cell apoptosis rate (Figures 6H,I). Taken together, LINC00320 can inhibit tumor growth and angiogenesis by upregulating AQP9.

**FIGURE 6:** LINC00320 overexpression inhibited tumor growth and angiogenesis through downregulation of AQP9. **(A)** Quantitative analysis of xenograft tumor volume in nude mice, *n* = 10. **(B)** Representative images of xenograft tumors excised from nude mice. **(C)** Quantitative analysis of tumor weight in mice, *n* = 10. **(D)** Protein band of VEGF protein in tumor tissues measured by Western blot analysis. **(E)** VEGF protein expression in tumor tissues normalized to GAPDH measured by Western blot analysis, *n* = 10. **(F)** CD31 protein expression identified by IHC assay (400×, scale bar = 25 μm). **(G)** IHC analysis of CD31 protein in nude mice, *n* = 10. **(H)** Cell apoptosis in tumor tissues identified by TUNEL assay (400×, scale bar = 25 μm). **(I)** Cell apoptosis rate in tumor tissues of each group, *n* = 10. *p < 0.05 vs. nude mice injected with U87 cells transfected with oe-NC. Data were expressed as mean ± standard deviation, and comparisons among multiple groups were conducted by one-way ANOVA, followed by Tukey *post hoc* test. The experiment was repeated three times independently.

## Discussion

Identified long non-coding RNAs have emerged as important regulators of many biological processes and molecular mechanisms of the development and progression of devastating brain tumors such as glioma and neuroblastoma (Malissovas et al., 2018; Pop et al., 2018). The present study was designed to explore the regulatory mechanism whereby LINC00320 mediated effects on AQP9 expression and to identify their roles in glioma cell tumorigenicity and angiogenesis. Our results indicate that LINC00320 elevated the expression of AQP9 through the TF NFKB1, thereby inhibiting the proliferation of glioma cells and angiogenesis of MVECs.

Our initial results showed that LINC00320 was downregulated in glioma tissues, and overexpression of LINC00320 inhibited glioma cell proliferation and angiogenesis. LINC00320 is specifically expressed in human brain, with notable high expression in cortical white matter (Mills et al., 2015). LINC00320 is reported to be among the differentially expressed lncRNAs in breast cancer, but its modulatory role in cancer progression is yet to be determined (Dong et al., 2019). Consistent with our findings, others have illustrated that LINC00320 acts as a tumor-suppressive lncRNA to inhibit glioma cell proliferation by downregulating β-catenin and TCF4 (Tian et al., 2019). Our study provides additional evidence that LINC00320 functions as a tumor suppressor in glioma through reducing AQP9 expression. Additionally, we found that overexpressed LINC00320 resulted in suppressed MVEC angiogenesis as evidenced by diminished expression of VEGF, CD31, MMP-2, and MMP-9. VEGF, which is normally expressed in endothelial cells (ECs), is known to harbor proangiogenic properties, such that antibodies against VEGF can block angiogenesis in malignancies (Melincovici et al., 2018). Largely in agreement with our present findings, CD31 expression is elevated in glioblastoma multiforme, which is highly suggestive of aberrant angiogenesis (Musumeci et al., 2015). Likewise, loss of VEGF, MMP-2, and MMP-9 has a correlation with the suppressed angiogenesis of human umbilical vein ECs in hepatocellular carcinoma (Zhang et al., 2018). Therefore, LINC00320 could function as an antioncogene in glioma by repressing glioma cell proliferation and MVEC angiogenesis.

We also observed in this study that AQP9 had high expression in glioma tissues. Previous work documented that AQP9 is expressed in astrocytes and catecholaminergic neurons and that AQP9 serves a pivotal role in brain energy metabolism (Badaut, 2010). Moreover, AQP9 has been shown to function as a tumor promoter or tumor suppressor in different cancers. For instance, Zhang et al. have reported that overexpression of AQP9 could inhibit invasion of hepatocellular carcinoma cells by inhibiting epithelial–mesenchymal transition (Li et al., 2016; Zhang et al., 2018). However, the mRNA expression of AQP9 is upregulated in breast cancer, and high AQP9 expression may be related to worse relapse-free survival in that disease (Zhu et al., 2019). Chen et al. (2016) have demonstrated that the expression of AQP9 is detectable in prostate cancer cells, whereas inhibition of its expression impedes their growth and promotes cell apoptosis through effects on the extracellular regulated protein kinase signaling pathway. AQP9 also functions as an oncogene in astrocytoma by facilitating cell invasion and motility via the AKT pathway (Lv et al., 2018). Moreover, AQP9 is expressed at a high level in the tumor progenitor population and tumor tissues, and its expression exhibits relationships with tumorigenesis of glioblastoma (Fossdal et al., 2012). In line with an increased level of AQP9 in most glioma cells, which was positively correlated with pathological grade in previous studies (Tan et al., 2008; Jelen et al., 2013), the present study confirmed an increased expression in glioma at a tissue level. More importantly, downregulation of AQP9 was observed to exert inhibitory effects on angiogenesis in our hands. Consistent with this finding, loss of AQP9 has been indicated to suppress brain angiogenesis in the hippocampus after intracranial hemorrhage, as observed in a mouse model (Ji et al., 2017). Therefore, we hypothesized that LINC00320 could inhibit the progression of glioma by reducing AQP9, which was confirmed by our experiments *in vitro* and *in vivo*. Of note, compromised proliferation through downregulation of AQP9 was observed in our study. Downregulation of AQPs in endothelial and malignant cells has been demonstrated to inhibit tumor growth and metastasis, thus holding a therapeutic potential for treatment of tumors (Ribatti et al., 2014). Overexpressed AQP9 has been suggested to trigger p21 upregulation and S-phase arrest in colorectal cancer (Huang et al., 2017). However, low expression of AQP9 has been identified in hepatocellular carcinoma as well (Peng et al., 2016), which calls for further exploration regarding the functional role of AQP9 in the context of glioma, as comparison of AQP9 expression in various organs is also of great importance to identify potential off-target effects of their inhibitors.

To analyze this relationship, we performed RIP, dual-luciferase reporter assays, and ChIP assays. Those assays explained that LINC00320 reduced the expression of AQP9 by inhibiting the recruitment of NFKB1 to the promoter region of AQP9. It has been reported previously that NF-κB regulates many genes involved in brain function (Edenberg et al., 2008). NFKB1 subunit is a critical modulator of NF-κB activity, while its knockout contributes to malignancy (Cartwright et al., 2016). LINC00526 suppresses glioma progression by forming a double-negative feedback loop with AXL, where NFKB1 binds to LINC00526 promoter and represses the transcription level of LINC00526 (Yan et al., 2019). In this study, we found that NFKB1 could bind to the promoter region of AQP9 and upregulated its expression, whereas LINC00320 blocked the recruitment of NFKB1 on the AQP9 promoter and thus inhibited AQP9 expression. Accordingly, we now consider the possibility that LINC00320 inhibits AQP9 via mediating NFKB1, thereby inhibiting the proliferation of glioma cells and angiogenesis of MVECs.

In conclusion, the present study demonstrates that upregulation of LINC00320 can reduce the expression of AQP9 and ultimately inhibit the proliferation of glioma cells and suppress tumor angiogenesis (Figure 7). LINC00320 may be a promising therapeutic target for glioma, pending a more comprehensive description of its effects in human disease and animal models.

**FIGURE 7:** LINC00320 downregulates AQP9 via inhibiting the recruitment of NFKB1 to the promoter region of AQP9, thereby preventing glioma progression.

## Data Availability Statement

The datasets presented in this study can be found in online repositories. The names of the repository/repositories and accession number(s) can be found in the article/ Supplementary Material.

## Ethics Statement

The current study was performed with the approval of the Clinical Trial Ethics Committee of North China University of Science and Technology Affiliated Hospital. All patients and their families in the experiment gave informed consent to the experiment and signed informed consent. The animal experiment was approved by the Experimental Animal Ethics Committee and strictly adhered to the principle to minimize the pain, suffering and discomfort to experimental animals.

## Author Contributions

LC, ZB, and XX: conceptualization and experimental design. XX and JL: experiments supervision. LC, DW, FZ, JZ, and YZ: experiments execution. LC, XX, and ZB: data analysis. LC and JL: writing – original draft preparation. ZB, XX, DW, FZ, JZ, JL, YZ, and LC: writing – review and editing. All authors contributed to the article and approved the submitted version.

## Conflict of Interest

The authors declare that the research was conducted in the absence of any commercial or financial relationships that could be construed as a potential conflict of interest.

## Footnotes

1 https://www.ncbi.nlm.nih.gov/geo/

2 http://bio-bigdata.hrbmu.edu.cn/LncMAP/index.jsp

3 http://jaspar.genereg.net/

## Supplementary Material

Supplementary Figure 1 Cell death rate after transfection detected by trypan blue staining (200×, scale bar = 50 μm).

## Abbreviations

AQP9: aquaporin 9
CCK-8: cell counting kit 8
LINC00320: long intergenic non-coding RNA 00320
lncRNAs: long non-coding RNAs
MVECs: microvascular endothelial cells
NFKB1: nuclear factor κ B subunit 1
ChIP: chromatin immunoprecipitation
RT-qPCR: reverse transcription–quantitative polymerase chain reaction
SPF: specific pathogen free.
